RETRACTED

# An Application for Measuring and Analyzing the Level of Performance Accuracy for Health Services Quality Indicators by Using Six-Sigma: A Study Case of Government Hospitals in Khartoum State

**DOI:** 10.1155/2021/8425206

**Published:** 2021-10-29

**Authors:** Amal Hassan Mohammed Yassin, Najla Elzein Abukassawi Osman, Wiem Abedelmonem Ben Khalifa, Eltahir Nouh Mohammed Adam

**Affiliations:** ^1^College of Arts, Imam Abdulrahman Bin Faisal University, Dammam, Saudi Arabia; ^2^College of Social Studies and Economics, University of Bahri, Khartoum, Sudan

## Abstract

The study aimed at acknowledging the Six Sigma methodology and the existence of the essential components for the application, as well as reducing the time for completing the operations, reducing the error rate to the lowest possible level, and improving the quality of operations. For this objective, the analytical descriptive methodology was used on a sample consisted of 300 administrative and medical staff from Khartoum State Hospitals (Khartoum, Omdurman, Bahri). To this end, a questionnaire was used for collecting data and for analyzing it and achieving the results of the study by using the statistical analysis package (SPSS). The study deduced a number of results, the most important of which are that the items of commitment and supreme command support for the senior leadership and the methods of abundant human resources on quality control, and the application of the Six Sigma methodology in government hospitals in Khartoum state achieved a satisfactory level, while continuous improvement paragraphs, processes, and systems on quality control and the application of Six Sigma methodology achieved high quality. There is a significant effect on the extent of commitment and support of the higher leadership on quality control and the application of the Six Sigma methodology. Similarly, there is a statistically significant effect on the application of continuous improvement methods on quality control and Six Sigma methodology. Also, there is a statistically significant effect on the application of the abundance of human resources methods variable on quality control and the application of Six Sigma methodology in governmental hospitals in Khartoum state. The study recommended to take interest in the Six Sigma methodology and assure the possibility of using it in Khartoum State's hospitals because of its scientific and practical importance in improving the quality of services and provided processes, and the need to provide qualified financial and human resources for using and developing Six Sigma methodology in hospitals, as well as great attention in training and providing departments heads with full knowledge of Six Sigma methodology and the fundamentals on which Six Sigma methodology, is based on its importance for hospitals. The study also recommended associating the promotions system in government hospitals in Khartoum state with the quality control program.

RETRACTED

## 1. Introduction

The purpose of applying Six Sigma methodology lies in performance monitoring, activities, business, and daily services to access the highest levels of quality, by reducing the percentage of waste and defective opportunities in a manner that meets customer needs. This methodology is considered a conceptual complex consisting of a statistical measure of performance related to operations, product manufacturing, and service provision. The Six Sigma methodology has been included into quality control in hospital work, performance monitoring, and health services to raise the level of these services and monitor them, in addition to leveraging and improving the provided processes and services.

The challenges and economic and financial variables that are facing global and local organizations, institutions, and sectors are embedded in increasing the competitiveness in the level of services they provide. It may be accompanied by a change in the consumer's behavior who has become more aware of the consumption culture and has a greater ability to select the best service after adopting quality as a basic criterion for choosing the services provided to the consumer.

Six Sigma indicates that the symbol *σ* is used to denote the standard deviation, which refers to the deviation, variation, or dispersion in a particular process in relation to the desired goals [1], and its historical background extends to more than eighty years starting from practical management principles developed in the United States in a major achievement to Japanese management in the 1970s [2].

Since Motorola launched Six Sigma in 1986, its spread has increased globally, as it began in the public sector, where he began to think about how he could benefit from this methodology and improve his performance.

Medical services are unique in their nature since any medical error in providing the service may threaten the life of a patient. Similarly, its techniques are various. Thus, it is not possible for the average citizen to verify the correctness of the decision himself. The nature of health services requires that the health care service be accompanied by a degree of certainty of its results, and this increases the advantages of the health care service. The health care organization that applies the concepts of Six Sigma has a high rate of errors, as well as the level of service can be predicted and confirmed.

RETRACTED

The problem of the study lies in the lack of training on the Six Sigma by the hospital administration, which, in turn, reduces the quality of the health services provided, the lack of awareness of the importance of this methodology and its role in improving health services, the disparity of the quality services provided among the hospitals of Khartoum state, and the lack of scrutiny and control for the application of the Six Sigma methodology to reach health care and reduce health service errors on many occasions.

The importance of the study stems from the importance of applying Six Sigma methodology and shedding light on concepts and the mechanism of applying this methodology to obtain results that are practically useful for hospitals. It is also useful for benefiting the study community from hospitals and health sectors. Also, research is useful in opening similar research fields to identify the importance of applying the Six Sigma methodology in quality control, especially in the health sector. The study also provided suggestions that benefit the study community, shedding light on weaknesses and enhancing the strength in the application of this methodology and its importance to health sector, Khartoum state hospitals, and their role in improving the provided health services.

The objectives of this study revolved around identifying Six Sigma methodology, steadily improving the quality of operations, reducing costs and developing them, reducing the time taken to complete operations, reducing the error rate to the lowest possible level, and identifying the availability of having the necessary components for the application.

The study adopted descriptive and inferential approaches by using practical study and attempting for applying Six Sigma on such a study.

Data related to this study were obtained by referring to literature, books, theses, scientific research, and journals in order to build the theoretical framework of the study and achieve its objectives. As for the study population, it is a case study for clarifying the possibility of applying Six Sigma methodology to government hospitals in Khartoum state (Khartoum, Omdurman, Bahri) and to examine the availability of the components of applying this methodology and its role in improving health services.

## 2. Theoretical Aspect

### 2.1. Concept of Six Sigma Methodology

#### 2.1.1. Sigma *σ*

It is the eighteenth letter in the Greek alphabet. Statisticians have used this letter to denote the standard deviation, which is considered as a statistical measurement and an indicator to describe the deviation, variance, or dispersion. The root of *σ* considered as a standard for measuring deviation can be traced back to Carl Frederick Gauss (1777–1855 AD) who introduced the concept of normal curve.

RETRACTED

#### 2.1.2. Standard Deviation

It is a statistical tool for measuring the extent of dispersion of (*Xi*) values from their means ($\bar{X}$).

The standard deviation expresses the extent of distance or dispersion from the mean which indicates an increase in the amount of error, which means an increase in product damage or a decrease in quality in providing service. Therefore, the Six Sigma methodology is considered as one of the important methods that aims at reducing the size of the error to the furthest extent, i.e., reducing the percentage of defects and errors to the minimum possible [3]^.^

However, number six symbolizes a level of sigma levels, where there are several levels of sigma, which of course represent several levels of quality. The more the number associated with sigma increases, this indicates an increase in the quality level and of course the decrease in the percentage of defects in the product, and vice versa. To clarify, the decrease in the number associated with sigma indicates the low level of quality, and there are certain sectors that use Eight Sigma instead of Six Sigma, such as the airlines sector and the ophthalmic medicine and surgery sector [4].

### 2.2. Among the Most Important Definitions of Six Sigma

- It is defined as “a statistical measure of processes and products, aiming to develop businesses with the fewest possible defects, and that it is a management system that seeks to achieve strong leadership by motivating and engaging members of the organization” [1].
- In another definition, “it is a letter in the Greek alphabet and it has become a statistical symbol indicating the standard deviation that it is used to measure the difference or deviation from the means” [5].
- It is also a statistical tool by which you can quantitatively measure the level of performance of one or more quality indicators by measuring the number of chances of defects precent in millions of DPMO (Defects Per Million Opportunities) [6].
- Six Sigma considers something different for every company, while for some people, it considers as a comprehensive management philosophy, and for others, it simply considers as efforts to improve processes designed to increase productivity and reduce costs [7].
- From the researcher's perspective, it is the method of implementation at the operating level in which the error does not exceed 3.4 chances per million, a statistical measure of error-free performance.

### 2.3. Organizational Structure of the Six Sigma Team

After the senior management in the facility decides to use Six Sigma methodology, it must begin to form a team consisting of leaders and members, and each has its function within this system. Each member of this team was given a name that refers back to the art of karate, which is an art of courage, such as The Master Black Belt, the Black Belt, and the Green Belt, and these names were invented by a Motorola expert who adores the art of karate.

RETRACTED

### 2.4. Principles of the Six Sigma Method

According to a previous study ((The Extent of Adherence to Six Sigma methodology) in Controlling the Quality of Internal Auditing - An Applied Study on Banks Operating in Gaza Strip - 2012 pp: 16-17) each of [4] referred to the basic principles on which the Six Sigma methodology is based on.

### 2.5. Genuine and Sincere Focus on Customer Satisfaction

Clients in the philosophy of Six Sigma methodology include customers and employees of the facility. The continuity and success of the facility depends on meeting their needs and expectations and trying to implement them. Customer's satisfaction is considered the main pillar in achieving quality. The Six Sigma methodology places the highest priorities to focus on customers, as it begins with studying the requirements and expectations of the customer and ends with studying the customer's satisfaction with the product or service.

### 2.6. Management Based on Facts and Data

The Six Sigma methodology helps the facility to obtain better data, as these establishments evaluate the performance by focusing on realistic and sufficient data that reflects customer requirements, containing costs and reducing defects. Realistically, the Six Sigma methodology helps managers answer two key questions to support decision-making and data-based solutions:

1. What data and information does the establishment really need?
2. How can we benefit from these data and facts to the maximum extent possible?

### 2.7. Focus on Internal Processes and Activities

When applying the Six Sigma methodology, every practical procedure constitutes a process in itself, whether it is a design of products and services, a measure of performance, improvement of effectiveness, or customer satisfaction. Therefore, we focus on the designed products, services provided, performance, customer satisfaction, and continuous improvement. Six Sigma sets the process as the main focus for the company for sustained success.

### 2.8. Effective Management Based on Advance Planning

It means that successful management seeks to address the problem before it occurs, i.e., there are administrative and technical measures that are taken before the problem occurs in order to avoid it.

### 2.9. Cooperate beyond Borders

The cooperation element is one of the vital elements that helps to achieve success and improve teamwork at all administrative levels of the company and with sales agents and customers. The Six Sigma methodology focuses on the importance of cooperation between the various administrative levels in the organization instead of competition between them. However, through cooperation, departments can know the needs of other departments in terms of financial and technical resources and other various requirements that help support the process of continuous improvement of the facility.

RETRACTED

### 2.10. Striving for Excellence with the Ability to Withstand Failure

Six Sigma emphasizes the importance of striving for excellent principle with the ability to withstand failure because the two ideas complemented each other, if people who strive for excellence in performance fear failure, they will never try. The essential point of this principle is that any firm that sets the six sigma methodology as its goal must continue to strive to strive for excellence in performance, while at the same time, it is amenable and able to manage some setbacks from time to time.

#### 2.10.1. Success Factors for Six Sigma Methodology [6]

The four primary factors for the success of the Six Sigma project are ranked according to their importance:

1. The support and participation from senior management
2. Allocating adequate resources to the improvement team
3. Decision-making driven by data, information, and facts
4. Measuring and taking appropriate corrective measures for the ruling factors in the process.

From the researcher's point of view, these factors must be interrelated and related to each other in order to ensure the success of the Six Sigma methodology as required.

#### 2.10.2. Determinants of Applying Six Sigma Methodology [8]

Some of the determinants of applying the Six Sigma methodology are as follows:

- The lack of data of the required quality, especially at the beginning of operations (the data collection phase may take a long time in the facility)
- The statistical definition of Six Sigma is 3.4 defect or failure per million opportunities in the industry sector that can be calculated, while in the service sector, anything that does not meet the needs or expectations of the customer is considered a failure or a mistake
- The choice and preference of projects still depend on personal decisions
- The change in the level of the Six Sigma methodology in services may not be significant
- The Six Sigma methodology can be easily bureaucratic due to the presence of black and green belts on which any project within the facility is based

#### 2.10.3. Some of the Determinants of Applying Six Sigma Methodology

Some of the determinants of applying the Six Sigma methodology are as follows:

- The lack of required quality data, especially at the beginning of operations (the data collection phase may take a long time in the facility).
- The statistical definition of Six Sigma is 3.4 defect or failure per million opportunities in the industry sector that can be calculated, while in the service sector, anything that does not meet the needs or expectations of the customer is considered a failure or a mistake
- The choice and preference of projects still depends on personal decisions
- The change in the level of the Six Sigma methodology in services may not be significant
- The Six Sigma methodology can be easily bureaucratic due to the presence of black and green belts on which any project within the facility is based

RETRACTED

### 2.11. Applying Six Sigma in Health Sector

According to a previous study (Six Sigma applications in the health field, Dina Ismail Al Kayyali, Master of Applied Statistics, Cairo University), the application of Six Sigma in health care is connected with the management of work policy and the strength of quality improvement than just the application of statistical methods in measurement. Healthcare institutions are inherently complex and have many overlaps between physicians, nurses, administrators, regulators, and consumer representatives who do not agree on a single method of change.

Since the environment is inclined to deny the error or at least conceal it with rational arguments, identifying common scorecards for measuring quality is considered a very important stage. It is worth noting that Six Sigma can measure performance by using general standards. Thus, we can determine the control of error and then monitor it. Six Sigma is defined as the process of analyzing technical processes to raise the level of quality of health care and services in line with patient requirements. Six Sigma focused on technical operations and the use of statistical methods to reduce medical errors, such as administering wrong medication in surgical operations and providing high-level services such as speed of entry or accounting errors. Six Sigma is also defined in the health sector as a systematic statistical process to detect and treat defects in performance by using Six Sigma methodology to reduce clinical and mechanical bottlenecks that lead to extended time, high costs, and poor results.

### 2.12. Previous Studies

1. [9]
2. This study aimed to identify the main components of Six Sigma in order to understand its strategic characteristics. Recently, SS has become one of the best tools for the healthcare system because it develops core competence in healthcare that deals with crucial needs in patient care and safety. This study applies LSS to improve the medical process of acute myocardial infarction. The defined measure analyzes, improves, and controls steps of SS, finds critical-to-quality factors, and draws the value stream map to seek out non-value-added activities. The cause and effect diagram is also employed to analyze the root causes of waste and generate the improved project by brainstorming. Eliminating waste raises the process cycle efficiency. The study results indicate that LSS not only improved medical quality but also strengthened market competitiveness.
3. Measuring the Quality of Health Services in Government Hospitals in Sudan from the Point of View of Patients and Auditors - A Field Study on Major Teaching Hospitals in the State of Khartoum (Mohammed Nour Al-Taher Ahmed Abdel-Qader, 2015):

Measuring the quality of services is one of the main entrances to improving and developing quality in service organizations. However, we find that there is a discrepancy in determining how service quality is measured and the factors and variables associated with it, especially in the field of health work, due to the different schools and concepts of quality. The need has emerged that government hospitals should deal with the concept of quality and pay attention to it when providing their services to their clients, especially with the opening of the door for the private sector to invest in providing health services. We find that government hospital administrations in Sudan face several questions when providing their services to patients and visitors. The study showed the following results:

- There is a full awareness among patients and auditors in Sudan of the levels required to be available in hospitals when providing health services
- Governmental hospitals do not have the necessary and necessary material supplies to provide health services
- Governmental hospitals do not have qualified cadres who prefer to work in the private health sector
- Feeling insecure about obtaining health services in government hospitals in a timely manner
- Feeling of insecurity and fear of not having the necessary medical prowess of good cadres and assistance when receiving health services in government hospitals
- Explain that most patients and auditors turn their financial circumstances away from their visits to private hospitals, and therefore, they have no choice but to visit government hospitals

RETRACTED

## 3. Application Aspect

### 3.1. Six Sigma Implementation Stages (DMAIC Model)

#### 3.1.1. The Purpose of the Project

Learn about the Six Sigma methodology and the availability of the necessary components for the application, steadily improving the quality of operations, reducing costs, reducing the time taken to complete operations, and reducing the error rate to the least possible. The steps related to the application of Six Sigma methodology (DMAIC model) can be summarized as follows:

(i) The first stage: define
Three government hospitals were selected from Khartoum state hospitals, namely, Khartoum, Omdurman, and Bahri. A statistical questionnaire was designed and distributed to the three hospitals; after it was presented to a number of arbitrators, the reliability and validity factor was confirmed by 320 questionnaires. 300 questionnaires were retrieved that can be statistically analyzed that accounted for 94%.
(ii) The second stage: measure
Data and information were collected from the sample members, as it is considered a representative statistical sample of the research community. After collecting the data, the statistical program SPSS (Statistical Package for Social Sciences) was used to extract the frequencies, percentages, and means. The results showed that 59% of the sample individuals did not receive training on Six Sigma.
A summary of what was observed and what was considered to be the cause of the delay was written, focusing on improvement opportunities, and then an action plan for improvement was prepared.
(iii) The third stage: analysis
Think of the problem like this:
  (1) $$\begin{array}{c} Y=f\cdot \left(X\right), \end{array}$$
where *Y* represents the goal of the project, which is to identify the Six Sigma methodology and *x* is the basic factor affecting the application of this methodology, which are four factors that were placed in the form of hypotheses where the *t*-test was used to test these hypotheses.
(iv) The fourth stage: improvement
  (a) Conducting educational brochures for employees of the Six Sigma methodology and its importance in quality control in hospitals
  (b) Conducting training courses on Six Sigma for administrators and those responsible for quality control in hospitals
  (c) Unlimited cooperation between the different departments of the concerned hospitals and linking them to an electronic network with the ministry.
  (d) Senior management awareness of the importance of Six Sigma and the need to apply it in hospitals to ensure the quality of operations, reduce error to the least possible, and reduce the time taken to complete various operations.
(v) Fifth stage: the control phase
To monitor the results, the study will be done after a period of time to ensure the improvement of the processes and to follow-up the progress towards the goal and take the necessary measures.

### 3.2. Tests Related to the Validity of the Instrument (the Questionnaire)

#### 3.2.1. Instrument Validity Study Tool

The virtual validity of the study tool was verified by presenting it to [7] of the arbitrators from the specialized professors.

RETRACTED

The necessary adjustments were made by modifying, canceling, or adding paragraphs of the questionnaire in a way that achieves a balance between the contents of the questionnaire in its paragraphs and to become more clear to the members of the study sample and more honest in measuring the required variables.

#### 3.2.2. Reliability Study Tool

To ensure the stability of the tool, the internal consistency factor (Cronbach's Alpha) was calculated (which is a single number and scale that measures the degree of reliability and validity of the questionnaire questions, i.e., the ability of the tool used in the research to measure its intended measurement). The Cronbach's Alpha coefficient, which is equal to (60%) at least, is an acceptable value to judge the validity of the research instrument or the questionnaire. The higher the value of the alpha coefficient, the greater the degree of reliability and validity between the questionnaire questions.

Cronbach's mathematical equation:

(2) $$\begin{array}{c} \alpha =\frac{N\cdot \bar{c}}{\bar{v}+\left(N-1\right)\cdot \bar{c}}, \end{array}$$

where

 
*N* represents the number of items
 
$\bar{c}$ represents the average interior contrast between the elements
 
$\bar{v}$ represents the mean total variance of the elements

### 3.3. The Statistical Methods Used in Data Processing

This study was based on the Statistical Package for Social Sciences (SPSS).

To carry out the statistical analysis of this study, the following statistical methods were used:

1. Frequencies and percentages to describe the characteristics of the study sample.
2. Internal consistency correlation Cronbach's alpha to check the stability of the instrument.
3. Means and standard deviations to answer the study questions.
4. *t*-test to verify the means related to the study questions.

The following Table 1 shows the values of Cronbach's Alpha coefficient for each axis of the resolution.

### 3.4. Defining the Levels of Responses

The researcher adopted Five-Point Likert scale to define the level of answers in the study tool, by placing a sign *x* for the answer that reflects the degree of their agreement, whether it is very high, high, medium, low, and very low. This is to assess the level of response to the study axes from the point of view of medical and administrative workers in government hospitals in Khartoum state. Three levels of means have been adopted as shown in Table 2.

### 3.5. The Description of the Characteristics of the Study Sample

The following tables show the frequencies and percentages of the study sample according to the demographic characteristics represented in age = *X*_1_, educational qualification = *X*_2_, total years of experience = *X*_3_, profession = *X*_4_, and the number of training courses they attended in the field of Six Sigma = *X*_5_.

RETRACTED

It is obvious from Table 3 and Figure 1 that the highest category is (41–50) that is achieved (144) by 48%, followed by the category (31–40) that is constituted (80) by 27%, while the lowest category (20–30) that achieved (76) with a percentage of 25%.

As shown from Table 4 and Figure 2 that workers achieved the highest category who possess bachelor's degree that accounted for (254) with a proportion of 85%, followed by workers who possess master's degree that amounted to (25) with the percentage of 8%, while the lowest category was for workers who have diploma or below, where their number reached (21) with the proportion of 7%.

As shown in Table 5 and Figure 3 workers occupied the highest category who have experience for 3 years or less as their number reached 230 with a percentage of 77%, while the lowest group was the share of workers who have experience from 4 to 5 years accounted for 70 with a percentage of 23%.

As shown in Table 6 and Figure 4, the highest category was the share of workers who are in the medical field, as their number reached 261, with a proportion of 87%, while the lowest group was the share of workers who are in the administrative field, as their number reached 39 with a percentage of 13%.

As shown in Table 7 and Figure 5, the highest category was for the workers who did not undergo training courses, as their number reached 178 with a percentage of 59%, followed by workers who have taken one course as their number reached 95 with a percentage of 32%, while the lowest category was for workers who have taken two courses that accounted for 27 with a percentage of 9%.

## 4. Findings and Discussion

### 4.1. The First Hypothesis

*H*_0_: there is no statistically significant impact for the commitment and support of senior management on quality control.

Table 8 and Figure 6 show that “the hospital administration has the necessary preparation to use Six Sigma methodology” with means accounted for 3.84, i.e., high quality, while the rest of the paragraphs achieved accepted means, indicating that the senior management has the necessary willingness to use the Six Sigma methodology. However, the financial and material capabilities of furniture, equipment, etc., and tools are limited. Likewise, you need to develop a solid strategic plan to properly implement the Six Sigma methodology (assessment according to table [10]).

Table 9 shows that null hypothesis was rejected while alternative hypothesis was accepted which indicates statistical significant difference at the statistical significance (*α* ≤ 0.05) the extent of commitment and support of senior management on quality control in Khartoum state in which the *t*-test value achieved 70.582 with a statistical significance of 0.00.

RETRACTED

### 4.2. The Second Hypothesis

*H*_0_: there is no statistical significance of continuous improvement on quality control and the application of the Six Sigma methodology.

Table 10 and Figure 7 indicate that all continuous improvement paragraphs are of high quality, which indicates that the government hospital administration in Khartoum state views continuous improvement as part of the quality requirements and for the purpose of reducing the deviations and errors that occur in the application of the Six Sigma methodology, as it relies on the Six Sigma methodology for the purpose of developing knowledge of dimensions of the administrative and technical process. It is also keen to know the customers' suggestions to benefit from them in improving the quality of services and training department heads to form working teams for the continuous improvement process. The hospital management also takes the necessary procedures to ensure that quality improvement plans are implemented by the employees.

It is obvious from Table 11 that null hypothesis *H*_0_ was rejected and the alternative hypothesis *H*_1_ was accepted, which indicates the existence of a statistically significant effect at the level of significance (*α* ≤ 0.05) in the application of continuous improvement methods on quality control and the application of six sigma methodology in governmental hospitals in Khartoum state. The value of *t*-test is 144.487 with statistical significance (0.00).

### 4.3. The Third Hypothesis

*H*_0_: there is no statistically significant impact on the abundance of human resources on quality control and the application of Six Sigma methodology.

As shown in Table 12 and Figure 8, it indicates that the hospital administration has the willingness and ability to appoint experts and consultants to implement the quality control program ....” It occupied the first rank with means achieved (3.76) with a high degree, which indicates that the hospital administration has a high willingness to appoint experts and consultants to implement the quality program, while the rest of the paragraphs were of an acceptable degree, such as linking promotions and rewards and assigning material and moral incentives to the application of quality control programs.

As shown in Table 13 that the null hypothesis *H*_0_ was rejected and the alternative hypothesis *H*_1_ was accepted, it indicates the existence of a statistically significant impact at the significance level (*α* ≤ 0.05) in the application of methods of the abundance of human resources on quality control and the application of Six Sigma methodology in Khartoum state hospitals, where the *t*-test value accounted for 82.154 with statistical significance (0, 00).

RETRACTED

### 4.4. The Fourth Hypothesis

*H*_0_: there is no statistically significant impact of processes and systems on quality control and the application of Six Sigma methodology.

As shown in Table 14 and Figure 9, the whole items achieved high-quality means, which indicates that the government hospital administration in Khartoum State is fully prepared to provide a system for exchanging information and its flow between quality control programs and direct contact with the trainers of these programs and providing a system for collecting information about patients and the services provided to them and update it on an ongoing basis, and the senior management has the possibility to provide software that enables the use of modern tools and techniques in the training process and the implementation of training programs on clear bases and standards.

As shown in Table 15, the null hypothesis H_0_ was rejected and the alternative hypothesis H_1_ was accepted, which indicates the existence of a statistically significant effect at the significance level (*α* ≤ 0.05) of both processes and systems of quality control and the application of Six Sigma methodology in Khartoum state hospitals, where the *t*-test value accounted for 123.105 with statistical significance (0.00).

It is obvious from Table 16 that the assessment of the means of the first hypothesis (senior management support) and the third hypothesis (the abundance of human resources) is accepted, while the assessment of the second hypothesis (continuous improvement) and the fourth hypothesis (processes and systems) achieved of high quality. This indicates that there is insufficient support from the senior management on quality control and the application of Six Sigma methodology in the three hospitals, as well as there is no necessary training to provide administrators and doctors with sufficient knowledge to use Six Sigma, while hospitals work on continuous improvement and have the processes and systems to apply the methodology.

## 5. Findings

The study came up with the following findings:

1. The highest category was for workers who possess a scientific qualification (bachelor's degree), as their number reached 254 with percentage 85%, and the second-highest number was for those who obtained a master's degree whose number reached 25 with percentage 8%; this indicates the presence of a good percentage of higher academic levels among the department directors in the government hospitals in Khartoum state.
2. There is insufficient commitment and support from the senior management to work on quality control and apply the Six Sigma methodology in Khartoum state hospitals, as a function of its general means, which has a value of 3.50 with an accepted assessment standard deviation of 0.86 and variation coefficient of 29%.
3. Lack of a clear strategic plan in implementing the Six Sigma methodology.
4. Hospitals are working on continuous improvement to work on quality control and the application of Six Sigma methodology in Khartoum state hospitals in terms of its general means, which has a value of 4.11 with a high quality evaluation, standard deviation of 0.49, and variation coefficient of 12%.
5. The study sample of medical and administrative workers agreed that the hospital administration is keen on training department heads to form work teams for the continuous improvement process to reduce the deviations and errors that occur in applying the Six Sigma methodology.
6. There is no abundance of human resources to work on quality control and the application Six Sigma methodology in Khartoum state hospitals in terms of its general means, which accounted for 3.39 with an accepted assessment, the standard deviation accounted for 0.72, and the coefficient of variation achieved 21%.
7. The hospital administration has the willingness and ability to appoint experts and consultants to implement a high-quality quality control program, while there was no preparation necessary to link promotions in the hospital to the quality control program.
8. The hospital administration has the processes and systems to work on quality control and the application of Six Sigma methodology in Khartoum state hospitals in terms of its general means, which has a value of 4.06 with a high quality evaluation, standard deviation accounted for 0.57, and coefficient of variation accounted for 14%.
9. The hospital administration is ready to provide an information system whose data are updated continuously.
10. The presence of a statistically significant impact in the application of continuous improvement methods on quality control and the application of Six Sigma methodology in governmental hospitals in Khartoum state.
11. The existence of a statistically significant impact in the application of methods of abundant human resources on quality control and the application of the Six Sigma approach in governmental hospitals of Khartoum state.
12. The presence of a statistically significant impact on the extent of commitment and support of the senior management on quality control and the application of Six Sigma methodology in government hospitals in Khartoum state. [11–13].

RETRACTED

## 6. Recommendations

In the light of findings that the study has come up with, the study recommended the following issues:

1. Emphasis is being given to Six Sigma and assuring the possibility of using it in Khartoum state hospitals due to its importance in both scientific and practical aspect, improving the quality of services and provided processes
2. The necessity of providing qualified human and financial resources for using and improving Six Sigma in the hospitals
3. The heightened interest in training and providing the department heads a complete knowledge of the Six Sigma methodology in the hospitals and the basics that underpin the Six Sigma methodology and its importance for hospitals
4. Connecting the promotion system in the government hospitals in Khartoum state with quality control program
5. Support and participation from senior management
6. Allocating the essential resources for the improvement group
7. Decision-making for data, information, and facts
8. Measuring and taking appropriate reform measures for the key elements in the process
9. Conducting further studies for indicating the impact of applying Six Sigma on other sectors
10. Conducting further studies after a period of time for indicating the impact of applying Six Sigma on quality control in the government hospitals in Khartoum state

## Figures and Tables

**Figure 1:** The distribution of age according to the study sample. Source: prepared by the researchers by using Excel 2017.

**Figure 2:** Academic qualification according to the study sample. Source: prepared by the researchers by using Excel 2017.

**Figure 3:** The years of experience according to the study sample. Source: prepared by the researchers by using Excel 2017.

**Figure 4:** The work field according to the study sample. Source: prepared by the researchers by using Excel 2017.

**Figure 5:** The number of courses that the sample attended in the Six Sigma field. Source: prepared by the researchers by using Excel 2017.

**Figure 6:** Findings of the commitment items and support of the senior administration assessment on quality control. Source: prepared by the researchers by using Excel 2017.

**Figure 7:** Findings of evaluating continuous improvement items on quality control. Source: prepared by the researchers by using Excel 2017.

**Figure 8:** Assessment results of the abundance of human resources items on quality control. Source: prepared by the researchers by using excel 2017.

**Figure 9:** Results of an evaluation of the operations and systems items on quality control.

RETRACTED

**Table 1:** Results of internal consistency coefficient (cronbach's alpha).

Axis	Alpha value	Intrinsic validity
First axis: the commitment and support of senior management and tools in quality control and the application of Six Sigma methodology.	0.90	0.95
Second axis: the continuous improvement in quality control and the application of Six Sigma methodology.	0.73	0.85
Third axis: the availability of processes and systems for applying Six Sigma methodology.	0.74	0.86
Fourth axis: the availability of human resources in quality control and the application of Six Sigma methodology.	0.76	0.87

Source: prepared by the researchers by using SPSS 26.

**Table 2:** Assessment according to the average.

Average	Assessment
Higher than 3.6	High quality
From 2.6 to 3.6	Accepted
Less than 2.6	Needs improvement

Source: prepared by the researchers by using SPSS 26.

**Table 3:** Respondents' age according to the study sample.

Age	No.	Frequency (%)
30–20	76	25
40–31	80	27
50–41	144	48
Total	300	100

Source: prepared by the researchers by using SPSS 26.

**Table 4:** Educational level according to the study sample.

Educational level	No.	Frequency (%)
Diploma or below	21	7
Bachelor	254	85
Masters	25	8
Total	300	100

Source: prepared by the researchers by using SPSS 26.

**Table 5:** Experience years according to the study sample.

Years of experience	No.	Frequency (%)
3 years or less	230	77
4-5 years	70	23
Total	300	100

Source: prepared by the researchers by using SPSS 26.

**Table 6:** Clarifies the work field according to the study sample.

Work field	No.	Frequency (%)
Medical	261	87
Administrative	39	13
Total	300	100

Source: prepared by the researchers by using SPSS 26.

**Table 7:** Number of training courses that the sample attended in Six Sigma methodology.

Training courses	No.	Frequency (%)
Nothing	178	59
One course	95	32
Two courses	27	9
Total	300	100

Source: prepared by the researcher by using SPSS 26.

**Table 8:** Means for the items of commitment and support of senior management on quality control.

No.	Items	Mean	Assessment
1	The hospital administration has the necessary preparation to use the Six Sigma methodology	3.84	High quality
2	The hospital administration has the financial ability to use the Six Sigma methodology	3.45	Accepted
3	The hospital administration has the financial means (furniture, equipment, ...) to use the Six Sigma methodology	3.49	Accepted
4	The hospital administration is ready to provide the facilities, time and tools for using the quality control program	3.47	Accepted
5	The administration has a clear strategic plan in applying the Six Sigma methodology	3.28	Accepted
Overall average		3.50	Accepted

Source: prepared by the researchers by using SPSS 26.

RETRACTED

**Table 9:** Results of applying one-sample *t*-test to measure the extent of commitment and support the senior management on quality control.

Field	Mean	Standard deviation	Degrees of freedom	*t*-test	Statistical significance
Measures the extent of commitment and support of the senior management to quality control in Khartoum state hospitals	3.50	0.86	299	70.582	0.00

Source: prepared by the researcher by using SPSS 26.

**Table 10:** Means of continuous improvement items on quality control.

No.	Items	Mean	Assessment
1	Hospital management considers continuous improvement as part of its quality requirements	4.06	High quality
2	Hospital management depends on the Six Sigma methodology for the purpose of developing the knowledge for the administrative and technical dimensions of the process	4.09	High quality
3	The hospital management is keen on knowing customers' suggestions to use them in improving the quality of services	4.13	High quality
4	The hospital management is keen on training department heads to form working teams for the continuous improvement process	4.14	High quality
5	The hospital management takes the necessary procedures to ensure that quality improvement plans are implemented by the staff	4.13	High quality
6	The hospital management works on continuous improvement in order to reduce the deviations and errors that occur in the application of six sigma methodology	4.14	High quality
	Overall average	4.11	High quality

Source: prepared by the researcher by using SPSS 26.

**Table 11:** Results of applying one-sample *t*-test to the general average for measuring the extent of applying continuous improvement methods to quality control.

Field	Mean	Standard deviation	Degrees of freedom	*t*-test	Statistical significance
It measures the extent of applying continuous improvement methods are applied on quality control and the application of six sigma methodology in Khartoum state hospital	4.11	0.49	299	144.487	0.00

Source: prepared by the researchers by using SPSS 26.

**Table 12:** Means of the abundant human resources methodologies on quality control.

No.	Items	Mean	Assessment
1	The hospital administration is willing to attribute promotions in the hospital to the quality control program	3.10	Accepted
2	The hospital administration is willing to attribute the rewards of the senior management to the successful implementation of quality control program	3.37	Accepted
3	The hospital administration has the willingness and ability to appoint experts and consultants to implement the quality control program	3.76	High quality
4	Hospital management provides financial incentives to scientists who take responsibility for implementing the quality control program	3.40	Accepted
5	The hospital administration provides moral incentives to scientists who take on the responsibility of implementing quality control program	3.35	Accepted
Overall average		3.39	Accepted

Source: prepared by the researchers by using SPSS26.

RETRACTED

**Table 13:** Results of applying one-sample *t*-test for measuring the extent of applying human resource abundance methods to quality control.

Field	Mean	Standard deviation	Degrees of freedom	*t*-test	Statistical significance
It measures the extent to which human resource abundance methods are applied to quality control and the application of six sigma in Khartoum state hospitals	3.39	0.72	299	82.154	0.00

Source: prepared by the researchers by using SPSS 26.

**Table 14:** Averages of operations and systems items on quality control.

No.	Items	Mean	Assessment
1	The hospital administration is ready to provide a system for exchanging and flowing information among quality control programs	4.02	High quality
2	The hospital administration has the ability to provide a system for collecting information about patients and the services provided to them	4.03	High quality
3	The hospital administration is ready to provide an information system whose data is updated continuously	4.11	High quality
4	The hospital administration is ready to provide a direct communication system with the trainers of quality control programs	4.01	High quality
5	The senior management has the possibility to provide software that enables the use of modern tools and techniques for use in the training process	4.04	High quality
6	The hospital administration carries out training programs based on clear foundations and standards	4.12	High quality
Overall average		4.06	High quality

Source: prepared by the researcher by using SPSS26.

**Table 15:** Results of applying *t*-test for (one-sample *t*-test) on the general average to measure the impact of processes and systems on quality control and applying the Six Sigma methodology in Khartoum state hospitals.

Field	Mean	Standard deviation	Degrees of freedom	*t*-test	Statistical significance
It measures the impact of processes and systems on quality control and the application of the Six Sigma methodology	4.06	0.57	299	123.105	0.00

Source: prepared by the researcher by using SPSS 26.

**Table 16:** A comparison among the four hypotheses.

Axis	Hypothesis	Mean	Assessment	Standard deviation	*t*-test
Senior management support	First	3.50	Accepted	0.86	70.582
Continuous improvement	Second	4.11	High quality	0.49	144.487
The abundance of human resources	Third	3.39	Accepted	0.72	82.154
Processes and systems	Fourth	4.06	High quality	0.57	123.105

Source: prepared by the researchers by using SPSS 26.

RETRACTED

## Data Availability

The results of study are available within the manuscript.

## References

[1] Bruce S (2006). Decorations: controversy and consensus. *Journal of Zoology*.

[2] Naime A., Wassoes M., Rateb (2008). *Achieving Accuracy in Management Feasibility (Six-Sigma)*.

[3] Antony J. I. (2004). Six sigma in the UK service organization results from A pilot survey. *Managerial Auditing Journal*.

[4] Brue G. (2015). *Six Sigma for Managers*.

[5] Pete Aka (2002). ASQ six sigma forum. *Six Sigma Forum Magazine*.

[6] Salet O. A. (2009). *Research for Obtaining a Membership Degree*.

[7] Berzekoub B. (2008). *Six-sigma for excellence in business field manager’s guide for supervising in projects and six sigma groups*.

[8] Salet O. (2010). *A Road Map to Six Sigma. Profitability, Continuity, and Growth*.

[9] Yeh H.-L., Lin C.-S., Su C.-T., Wang P.-C. (2011). Applying lean six sigma to improve healthcare: an empirical study. *African Journal of Business Management*.

[10] Al Ayashy Z., Buaweesh S. (2019). *Using Six Sigma to Measure the Quality of Performance*.

[11] Tawfeeq M. A., Mhusan A. (2005-2006). *New Trends in Evaluation and Excellence in Performance,*.

[12] Pande P., Holpp L. (2002). What Is Six Sigma?.

[13] Park S. H. (2003). *Six Sigma for Quality and Promotion*.

